The article "Chemical Structures and Pharmacological Properties of Typical Bioflavonoids in Polygonati Rhizoma (PGR)" was retracted in 2023. Reasons: unreliable results or conclusions; concerns about the data; concerns about the peer review; concerns about the citations.

# Chemical Structures and Pharmacological Properties of Typical Bioflavonoids in *Polygonati Rhizoma* (PGR)

**DOI:** 10.1155/2022/4649614

**Published:** 2022-09-20

**Authors:** Min Luo, Zongren Hu, Zixuan Zhong, Lumei Liu, Chengxiong Lin, Qinghu He

**Affiliations:** ^1^Department of Rehabilitation Medicine and Health Care, Hunan University of Medicine, Huaihua, 418000 Hunan Province, China; ^2^Institute of 5G Health Management with Synergy of Chinese and Western Medicine, Hunan University of Medicine, Huaihua, 418000 Hunan Province, China; ^3^Department of Nephrology, The Second Xiangya Hospital, Changsha, 410011 Hunan Province, China; ^4^College of Integrated Traditional Chinese and Western Medicine, Hunan University of Chinese Medicine, Changsha, Changsha, 410208 Hunan Province, China; ^5^Huairen Hospital of Traditional Chinese Medicine, Huaihua, 418099 Hunan Province, China

## Abstract

Most medicines are coming with toxic and detrimental side effects. In addition, microbials are resisting the medicine. Therefore, alternative drugs with low toxic and side effects and low microbial resistance are needed. Plants offer good potential candidates due to a broad range of chemicals they contain. These chemicals have been studied, and research is still going on to probe chemical properties of plant chemicals. In China, traditional Chinese medicine is practised, whereby plant extracts are obtained, and then sold in packages for reasons like memory enhancement, cancer treatment, boosting immune system, and so on. Among the herbs cultivated in China is *Polygonati rhizoma* (PGR). This plant contains various bioflavonoids such as diosgenin, kaempferol, catechin, daidzein, and 3′-methoxydaidzein. In this review, we discussed the pharmacological effects of these chemicals, including luteolin antimicrobial activity in a manner that it circumvents antibiotic resistance; rutin antivenom property; kaempferol as an agent that mitigates neuropathic pain; genistein anticancer property; isorhamnetin's ability to alleviate chronic obstructive pulmonary diseases (COPD); proanthocyanidins' ability to deal with diabetic neuropathy and analgesic property of catechin.

## 1. Introduction

Plant secondary metabolites serve as a defence system that protects plants from physical, chemical, and biological attacks. More often, such chemical components are referred to as natural products. It is known that these chemical components do have a broad spectrum of therapeutic effects. Research on natural products has therefore been one of the major scientific endeavours [1].

Pei et al. [2] points out that traditional Chinese medicine is over 3000 years old, and it focuses on aspects like multiple pathways, multiple targets, and multiple components*. Polygonati Rhizoma* (PGR) is one of the Chinese traditional herbs and is known for having antihypertensive, anti-inflammation, anticancer, cardioprotective, and neuroprotective effects. It is also reported that the herb treats Alzheimer's disease (AZ). Research has found that the herb improves memory and learning abilities of AZ mice [3]. This paper serves to discuss on a few bioflavonoids in *Polygonati rhizoma* and their medicinal properties. The chemical substances discussed in this review were luteolin, rutin, rutin succinate, kaempferol, genistein, catechin, proanthocyanidin, and isorhamnetin.

The article "Chemical Structures and Pharmacological Properties of Typical Bioflavonoids in Polygonati Rhizoma (PGR)" was retracted in 2023. Reasons: unreliable results or conclusions; concerns about the data; concerns about the peer review; concerns about the citations.

## 2. Flavonoids in PGR

Wang et al. [4] named three of the flavonoids found in PGR which are rutin, syringetin-3-O-glycoside, and isorhamnetin (Figure 1). Scientists extracted 10 chemical components from 10 sections of PGR. The list is endless. Some records indicate that 7-hydroxy-2-(4-hydroxyphenyl)-chroman-4-one (DFV), diosgenin, sitosterol, *β*-sitosterol, baicalein, methylprotodioscin, 3′-methoxydaidzein, (2R)-7-hydroxy-2-(4-hydroxyphenyl) chroman-4-one, and (+)-Syringaresinol-O-beta-D-glucoside are other flavonoids contained in the PGR [5]. The purpose of this review article is to summarize and discuss several main bioflavonoids contained in PGR and their pharmacological effects.

### 2.1. Luteolin

Guo et al. [6] observed that luteolin ‘chelates' streptolysin O toxin inhibits its cytotoxicity and haemolytic effects. Group A *Streptococcus* (GPAS) bacteria produce the aforementioned toxin and cause a wide range of diseases. Multidrug resistance (MDR) is persisting. As a result, herbal medicine is chipping in as one of the ways to circumvent the MDR [7]. Luteolin (Figure 2) has an antibacterial activity [8]. According to Zhang et al. [9], luteolin circumvents antibiotic resistance in *Trueperella pyogenes*. Scientists aim at the virulent part of pathogenic bacteria. In most cases, this virulence moiety is a toxin, which is a hemolysin-like protein. This approach is also another attempt to “bypass” antibiotic resistance [10].

#### 2.1.1. Luteolin and Streptolysin O (SPO) Toxin

According to Guo et al. [6], luteolin inhibits SPO haemolytic effect. The team adopted the erythrocyte homolytic assay reported by Dong et al. [11] and Dong et al. [12]. Previous research had reported that luteolin achieved anti-group A *Streptococcus* activity with the (minimal inhibit concentration) MIC of 128 *μ*g/mL. Guo et al. reported a lower MIC. The research team went on to analyze interaction between luteolin and SPO. The methodologies used were molecular docking and molecular dynamics (MD) simulations. Howbeit, Morra et al. [13] said that MD simulations are better than molecular docking. It was observed that luteolin binds SPO domains 1 and 3. The domains were characterised by *β* pleats hedged both sides by helices. The binding site is deemed to be a semiopen hydrophilic binding site. A magnitude of −7.2 kcal/mol binding energy was computed following luteolin-SPO interaction. Hydrogen bonds, van der Waals' forces, and hydrophobic interactions were the main forces involved during luteolin-SPO interaction. Tyrosine residues, glycine, aspartate, and isoleucine were the amino acids involved in luteolin-SPO interaction. Tyrosine residues were dominating the rest.

The article "Chemical Structures and Pharmacological Properties of Typical Bioflavonoids in Polygonati Rhizoma (PGR)" was retracted in 2023. Reasons: unreliable results or conclusions; concerns about the data; concerns about the peer review; concerns about the citations.

Guo et al. went further to make use of the MD simulations to comprehend the mechanism of the luteolin-SPO interaction. Conformational changes in SPO were found to be fluctuating. However, fluctuations were minimum when luteolin was bound to the SPO as compared to SPO alone. Therefore, the inference was that, luteolin stabilises the SPO conformation. No side-chain conformation was observed before or after luteolin-SPO interaction, which might help maintain the conformational stability of SPO and thus inhibit toxin assembly [6].

### 2.2. Rutin and Rutin Succinate

Rutin and its derivatives are part and parcel of the polyphenols called flavonoids. Rutin has the characteristics of bioavailability and solubility, which has not been studied in depth, which is a great challenge. Notwithstanding, rutin analogues were used instead to try and overcome bioavailability and solubility issues. Either natural or artificial rutin analogues can be used to understand pharmacological effects of rutin. Analogues like troxerutin and isoquercetin are useful. Artificially, rutin can be modified by adding succinate moieties on glycoside hydroxyl groups of rutin (Figure 1). Alternatively, metal ions can be conjugated to rutin [14].

#### 2.2.1. Rutin, Rutin Succinate, and Snake Venom

Snakebites are complex to treat. It has been a custom to treat snakebites by antivenoms from animals. As an illustration, *Bothrops* antivenom is used to treat individuals bitten by *Bothrops* snakes. Nonetheless, the incapacity to block local-induced snakebite effects and after-bite complications like oxidative stress is reported. Polyphenols, therefore, are a rightful candidate for snake venom treatment since they exhibit antioxidant properties. Research was done by Sachetto et al. where rutin succinate was tested for antivenom properties [14].

Sachetto et al. observed that rutin succinate has the ability to inhibit *Bothrops jararaca* (viper) venom *in vitro.* Rutin succinate inhibits of *Bothrops jararaca*'s hyaluronidase enzyme activity. The inhibitory effect varies with the inhibitor concentration. Other proteins of the viper venom (VV) were studied. These include venom metalloproteinases (VVMPs) and venom serine proteinases (VVSPs). Based on the findings of the research team, the inhibition rate of VVSPs inhibitors (which the research team called AEBSF) was 99.4%. VV activation of coagulation factors is one of the challenges to be addressed after snake bites. In vitro studies have shown that VV causes coagulation. Sachetto et al. analyzed the effect of VV on prothrombin activation. The team preincubated VV with rutin succinate and found that prothrombin activation was reduced by 98%, which greatly reduced the probability and degree of coagulation and also had a large positive effect on the treatment of snake venom [14]. Rutin succinate is expected to be a natural drug replacing specific inhibitors.

The article "Chemical Structures and Pharmacological Properties of Typical Bioflavonoids in Polygonati Rhizoma (PGR)" was retracted in 2023. Reasons: unreliable results or conclusions; concerns about the data; concerns about the peer review; concerns about the citations.

#### 2.2.2. Rutin and Rutin Succinate Silence VV Toxic Effects and Lethality

Sachetto et al. probed survival analysis of mice following administering the VV via intraperitoneal route. Two different doses were prepared. The first dose was twice lethal dose 50 (2LD_50_) and the second dose was thrice lethal dose 50 (3LD_50_). In their study, the first dose was used to induce envenomation. They then determined homeostatic parameters using the first dose. Severity of the venom was studied using the second dose. Incubation of rutin and rutin succinate was done with VV doses to observe the antivenom properties of the bioflavonoids, rutin, and rutin succinate.

In a space of 48 h, the first dose did not potentiate death in mice. According to their haematologic observations, incubating VV with rutin succinate mitigated leukocyte circulation in comparison with the VV alone mice group. The statistical *p* value for this result was less than 0.05. In the VV alone group, erythrocyte parameters were decreased by a range of 44-58%. This was not the case with VV + rutin succinate group. The inference is that rutin succinate prohibited a fall in erythrocyte parameters. The VV perturbed homeostatic balance causing hypofibrigenemia and thrombocytopenia. The experimental mice groups had lower platelets than normal following VV administration. It was found out that platelets dropped down to 53-86% below the expected platelet count.

The severe VV dose killed 50% of the mice in a space of 4 h. Other mice groups survived. After 48 h, the survival rate of 3LD_50_ alone group was 33.3%. It then follows that rutin succinate prohibits lethality of mice following VV administration [14].

### 2.3. Kaempferol

Kaempferol (Figure 3) was discovered in 1930. A Hungarian scientist by the name Albert Szent Györgyti managed to isolate a new chemical from oranges and it was believed to be one of the vitamins. Albert was a professor at the University of Szeged. It was then discovered that kaempferol is a flavonoid found in a broad spectrum of plants including Chinese plants like *Polygonati rhizoma* [2, 15].

The article "Chemical Structures and Pharmacological Properties of Typical Bioflavonoids in Polygonati Rhizoma (PGR)" was retracted in 2023. Reasons: unreliable results or conclusions; concerns about the data; concerns about the peer review; concerns about the citations.

#### 2.3.1. Kaempferol and Its Central Nervous System (CNS) Therapeutic Effects

In recent studies, kaempferol and its derivatives have pharmacological effects on a number of degenerative diseases like glioblastoma, Alzheimer, epilepsy, Parkinson, neuropathic pain, ischemic stroke, major depressive disorder, and anxiety disorders. These ailments are known for interfering with the nervous system [15].

#### 2.3.2. Neuropathic Pain and Kaempferol

The International Association for the Study of Pain defines neuropathic pain (neuralgia) as the nervous system pain generated when dysfunction and or abrasion of the nervous system occurs. A plethora of factors destroy nerves and thus resulting in neuropathic pain. Ailments like strokes, multiple sclerosis, cancer, herpes zoster, and diabetic neuropathy can cause neuropathic pain. This disease is generally divided into two categories, mononeuropathy and polyneuropathy. Mononeuropathy is the damage of the single nervous pathway; whereas polyneuropathy is characterised by damage of numerous nerves and the pain is generalised and well located [16].

According to [15] best knowledge, there is not an article of late that reported isolation of kaempferol to carry out experiments and see if it treats neuropathic pain. Nonetheless, some studies assessed total kaempferol extracts that contained kaempferol [17]. In one of those studies, kaempferol exerted hypoglycaemic effect in diabetes mellitus animal models. It then implies that antioxidant activity of kaempferol prevented oxidative damage, thus, avoiding neuropathic pain [17].

#### 2.3.3. Kaempferol and Major Depressive Disorder

The World Health Organisation (WHO) defines major depressive disorder (MDD) as a mental health disorder that is characterised by loss of interest in pleasurable activities, incapacity to carry out daily routine activities for at least a fortnight, and tenacious sadness. The common symptoms accompanied by the ailment are suicidal thoughts, loss of determination, and thoughts to harm self. Tetracyclic antidepressants treat MDD. The drugs work by blocking receptors of neurotransmitters like dopamine, serotonin, and norepinephrine. The monoamine oxidase inhibitor depressants (MAOIs) interfere with the activity of monoamine oxidase enzyme hence escalating the CNS dopaminergic, serotonergic, and noradrenergic neurotransmitters. Stroke, hypertension, and heart attack are reported fatal results if the MAOIs are taken with food which is rich in tyramine. The food includes cheese and fermented food products [18].

The article "Chemical Structures and Pharmacological Properties of Typical Bioflavonoids in Polygonati Rhizoma (PGR)" was retracted in 2023. Reasons: unreliable results or conclusions; concerns about the data; concerns about the peer review; concerns about the citations.

To rectify the challenges, scientists had to look for alternatives. Such alternatives must deal with any of the transduction or endocrinological pathways that lead to MMD. Reports say that neuroinflammation and oxidative stress trigger MDD pathophysiology. Gao et al. [19] reported that kaempferol exhibits antidepressant effect due to its antioxidant capacity. Also, kaempferol exerted anti-inflammatory properties which were achieved via escalating prefrontal cortex AKT (serine/threonine kinase)/*β*-catenin cascade. The team assessed the antidepressant effects of narirutin flavonoids and kaempferol-3-O-glycoside (K3G) using female wild Wistar rats. The team designed their experiment in a manner that five groups of Wistar were given different obesogenic diets. There was a group which got 30 mg/kg body weight and K3G three weeks prior to mating. The rest of the groups were regimented to their respective diets till they reproduce and begin to lactate. According to the results of Gao et al., too much caloric diets during perinatal periods have the potential to escalate behavioural changes in animal models and humans. The group supplemented with K3G and narirutin did not suffer from depression.

### 2.4. Genistein

Genistein (Figure 4) is an isoflavonoid found in plants as well. The chemical is known for having anticancer properties particularly cancer that results following radiation exposure. It is reported that genistein protects the DNA from radiation damage by hunting for radicals generated. A number of experiments revealed that mice which were exposed to radiation did not develop cancer following genistein administration [20].

Zhang et al. [20] designed an experiment to investigate the anticancer potency of genistein on irradiated IEC-6 cells. The team discovered that cell apoptosis induced by radiation was mitigated by genistein. Also, gastrointestinal injury by ionizing radiation was found to be improved.

### 2.5. Proanthocyanidins

Proanthocyanidins (PACs) are oligomers of flavonoids. These chemicals can be described as condensed tannins which are gallic acid and catechin derivatives. It is known that PACs are made up of prodelphinidins, procyanidins, and propelargonidins. The PACs recently drew a lot of scientists' attention due to their antihyperglycaemic, antioxidant, anti-inflammatory, and anticell death properties [21]. Gong et al. [22] conducted an experiment to probe PACs' ability to treat diabetic neuropathy induced by cadmium.

#### 2.5.1. PACs and Glucolipid Metabolism

Gao et al. investigated the effects of PACs in diabetic neuropathy mice, induced by cadmium exposure. The fasting blood glucose (FBG) was determined during the entire course of their study. The FBG levels in different groups were higher than the normal accepted range. The group treated with PACs had shown a decrease in FBG levels thus indicating the potency of PACs in lowering FBG levels. Further biochemical parameters like plasma triglycerides (TG) content, total cholesterol (TC), low-density lipoprotein-C (LDL-C), and high-density lipoprotein-C (HDL-C) among others. It was then found that in diabetic neuropathy (DP) mice, TD, TC, and LDL-C levels decreased in comparison with the control groups.

The article "Chemical Structures and Pharmacological Properties of Typical Bioflavonoids in Polygonati Rhizoma (PGR)" was retracted in 2023. Reasons: unreliable results or conclusions; concerns about the data; concerns about the peer review; concerns about the citations.

#### 2.5.2. Effects of PACs on Transduction Pathway

Gao et al. further probed the effects of PACs on Keap1/Nrf2 and p38 MAPK pathways in relation to oxidative stress. Western blotting technology was employed to carry out this investigation. Expression of proteins involved in p38 MAPK and Keap1/Nrf2 pathways was done. It was then found that MAPK and p38 were expressed significantly in diabetes neuropathy mice. Nonetheless, upon PACs administration, the protein expression dropped.

Nrf2 expression decreased markedly whereas Keap1 levels escalated in diabetes neuropathy mice group. Upon treating the mice with PACs, Nrf2, and Keap1 expression levels reversed. Therefore, the inference is that PACs protect the diabetic neuropathy mice from harm by a mechanism that involves p38 MAPK and Keap1/Nrf2 transduction pathways [19].

### 2.6. Catechin and Neuropathic Pain

According to Foudah et al. [23], chronic constriction injury causes neuropathic pain development in Sprague-Dawley rats. The team used a neutral plate to evaluate spontaneous pain in rats. Catechin lessened the pain. A parameter known as motor nerve conduction velocity was determined to see if catechin had an effect. The research team observed catechin improved motor nerve conduction velocity in mice. Chronic constriction injury had resulted in loss of motor nerve conduction.

#### 2.6.1. Catechin and Nuclear Factor-Kappa Beta (NF-*κβ*)

Chronic constriction rats had an elevated level of DNA binding activity of NF-*κβ* in sciatic nerve cells. The DNA-NF-*κβ* binding activity decreased following catechin administration. Nociceptive response is related to the NF-*κβ* activation. Escalation of NF-*κβ* activation is linked with an improvement in nociceptive response. Increased inflammatory response results in pain. Inflammatory cytokine production increases during inflammation and pain. A reduction in pain that depended on catechin concentration was reported [23].

### 2.7. Isorhamnetin and Chronic Obstructive Pulmonary Disease (COPD)

Brandsma et al. [24] said that COPD is a severe disease that causes inflammation of the lungs resulting in narrow airways. The disease can lead to emphysema. The disease is treated with bronchodilators and corticosteroids. The COPD patients are insensitive to corticosteroids according to some research. Therefore, alternative anti-inflammatory therapy is needed. Plant-derived chemical are suitable for treating COPD due to the anti-inflammatory properties [25]. A recent study shows that isorhamnetin (Figure 5) relieves inflammation of the respiratory system [26].

The article "Chemical Structures and Pharmacological Properties of Typical Bioflavonoids in Polygonati Rhizoma (PGR)" was retracted in 2023. Reasons: unreliable results or conclusions; concerns about the data; concerns about the peer review; concerns about the citations.

#### 2.7.1. Isorhamnetin Pharmacological Effect in COPD Animal Models

In mice, isorhamnetin (IHN) improves cigarette smoke-induced COPD. Xu et al. [26] administered lipopolysaccharides in mice via intratracheal inhalation route two times. Mice were also exposed to cigarette smoke. These treatments led to the manifestations of typical COPD clinical symptoms. Erythrocytes increased in cigarette smoke-induced COPD. A decrease in the number of red blood cells was observed following administration of isorhamnetin.

It is known that COPD inflammation results in deposition of collagen fibres surrounding the airway. Consequently, lung tissue elasticity is mitigated, and COPD is worsened [27]. Cigarette smoke-induced fibrosis was probed by staining lung tissues sections with Masson trichrome. The control tissue had a very thin layer of collagen deposit. The cigarette smoke group resulted in thick layer of collagen around bronchioles and vessels. The layer diminished in the isorhamnetin + cigarette smoke group [26].

#### 2.7.2. Isorhamnetin Mode of Action in Treating COPD

The major pathway underlying inflammation is Nrf 2/Keap 1 [28]. Xu et al. [26] determined superoxide dismutase enzymes (SOD)1 and 2; Nrf 2 and heme oxygenase 1. Isorhamnetin enhances the expression of the above-mentioned proteins. This expression depended on the dosage of isorhamnetin. At low concentration (30 mg/kg), isorhamnetin did not enhance the expression of heme oxygenase 1. The research team observed that after isorhamnetin treatment, Keap 1 was down regulated, Keap 1 as the feedback regulator of Nrf 2. In addition, a protein known as p 62 controls the Nrf 2/Keap 1 pathway. The protein interacts with the Keap 1 directly leading to the disintegration of the Keap1 via ubiquitination [29]. Isorhamnetin promoted p62 accumulation thus Keap 1 disintegration [26].

## 3. Conclusion

Synthetic drugs have many side effects, and scientists are gradually turning their research back to natural products. Flavonoids are one of the natural products of interest. *Polygonati rhizoma* contains many flavonoids and has been used in many parts of the world. In this paper, some typical chemical substances contained in seminal vesicles were reviewed, including luteolin, rutin, kaempferol, genistein, proanthocyanidins, and isorhamnetin, and their typical pharmacological activities were also described, showing antimicrobial, anticancer, antioxidant, anti-inflammatory, and anti-snake venom properties. These active natural chemicals contained in the yellow spirit are expected to replace synthetic drugs as new research targets for disease treatment.

The article "Chemical Structures and Pharmacological Properties of Typical Bioflavonoids in Polygonati Rhizoma (PGR)" was retracted in 2023. Reasons: unreliable results or conclusions; concerns about the data; concerns about the peer review; concerns about the citations.

## Figures and Tables

**Figure 1:** Some flavonoids contained in PGR.

**Figure 2:** Chemical structure of luteolin.

**Figure 3:** The chemical structure of kaempferol.

**Figure 4:** Genistein structure.

**Figure 5:** Chemical structure of isorhamnetin.

## Data Availability

The data used to support the findings of this study are included within the article.
